The article "Characterization and Combustion Behavior of Single-Use Masks Used during COVID-19 Pandemic" was published in 2021. Journal: Materials (Basel).

# Characterization and Combustion Behavior of Single-Use Masks Used during COVID-19 Pandemic

**DOI:** 10.3390/ma14133501

**Published:** 2021-06-23

**Authors:** Ewa Maria Szefer, Tomasz Mariusz Majka, Krzysztof Pielichowski

**Affiliations:** Department of Chemistry and Technology of Polymers, Cracow University of Technology, 24 Warszawska St., 31-155 Cracow, Poland; tomasz.majka@pk.edu.pl (T.M.M.); kpielich@pk.edu.pl (K.P.)

**Keywords:** COVID-19, disposable plastic waste, face mask, thermal degradation, pyrolysis

## Abstract

This work aims to study the thermal degradation and combustion behavior of single-use masks commonly used during the COVID-19 pandemic. The sudden increase in plastic waste underlines the crucial need for a proper disposal method. Therefore, to develop a suitable method of thermal disposal, it is first necessary to identify the primary waste materials and then study their thermal and flammability behaviors using thermal analysis methods. This research focuses on the characterization of individual parts of the masks, their thermal degradation, and pyrolysis processes via FTIR, TG, and MCC analyses. FTIR analysis indicated that all three masks were made out of polypropylene sheets, while two of the ear straps contained polyamide 6. One of the samples was composed mainly of poly (ethylene terephthalate) fiber and thin inner EPDM rubber. The EPDM ear strap left the highest residue and showed the lowest flammability among all samples. The analysis of heat of combustion and thermogravimetry shows that the most heat is generated above 450 °C. Therefore, for the disposal of single-use masks to be effective, it should be carried out in the temperature range from 450 to 750 °C.

## 1. Introduction

A novel, highly contagious coronavirus SARS-CoV-2 (severe acute respiratory syndrome-coronavirus 2), known as COVID-19, emerged in December 2019, leading in a short time to a global pandemic that has posed a significant threat and challenge to world health and the economy [1]. The primary way of coronavirus transmission is the droplet route [2]. In addition, the new coronavirus is more contagious than influenza, as it has been confirmed that an infected person can transmit the virus without displaying any apparent symptoms [3]. Regrettably, the pandemic has thus far resulted in around 160,502,000 infected people and contributed to the deaths of 3,335,000 [4]. Under these circumstances, most countries in the world sanctioned regulations to prevent the spread of the infection, involving social distancing, the lockdown of restaurants and schools, and restriction of travel and outdoor activities. An essential line of defense against infection is physically limiting the spread of respiratory droplets and their contact with other people. This necessitates the use of personal protective equipment (PPE) like facemasks, gloves, and protective gowns. Because of this, the demand for these goods significantly increased in 2020 due to the expansion of COVID-19. Huge amounts of PPE used every day in most of countries in the world require establishment of disposal routes to reduce the harmful effects of their waste on the environment [5].

Single-use masks are produced mostly using non-woven tissues, generally made up of three or four thin layers and filtering around 85% to 99% of particles with dimensions higher than a micron [6]. The first layer of the sheet absorbs moisture, the second acts as a filter for infection agents, and the outer layer is a repellent for liquids [7]. The masks equipped with FFP2 or FFP3 filters are referred to as high-performance filtering masks [8]. In these masks, filtration is achieved by combining a web of polypropylene microfibers and electrostatic charge.

Despite the fact that there are plenty of biopolymers available on the market, most single-use masks and their packaging are made of fossil-derived polymers [9,10]. The standard textile used to mass-produce face masks is polypropylene sheets, made using spun-bond or melt-blown technology [6]. The spun-bond process is a non-woven manufacturing system that combines the spinning process with the sheet formation process by placing the bonding device in the same continuous line [11]. Despite the fact that there are plenty of biopolymers available on the market, most single-use masks and their packaging are made of fossil-derived polymers [8]. 

On the other hand, melt-blown non-wovens are considered the mainstream fibrous air filters because of their developed surface area, high barrier properties, narrow pores, and excellent overall porosity [12,13]. For example, electret melt-blown filters are promising materials for intensive filtration by electrostatic force, thanks to their advantageous capacities of storing abundant charges and creating a quasi-permanent electric field on the periphery of their fibers [14]. Nevertheless, as a result of bulk and surface conductivity, it is unavoidable that the electrostatic charge will decrease over time, which causes a significant reduction in filtration efficiency [15].

Apart from polypropylene, other commonly used polymers like polystyrene, polyethylene, or polyesters are suitable for manufacturing surgical face masks. Apart from fiber selection, the filtration efficiency of single-use face masks depends on the method of manufacture, the structure of the web, the cross-sectional shape of the fiber, and its change [16]. The non-woven technology ensures improved barrier properties as compared to cotton [6]. Furthermore, the use of disposable masks decreases the risk of contamination as compared to reusable ones. However, material recycling of used mask products is impossible, as they are frequently pathogen-contaminated and have to be handled as hazardous waste. Therefore, thermal utilization through the thermo-chemical process offers a reliable disposal route for used masks [17,18,19]. Understanding the reaction mechanisms in the face mask plastic waste thermal degradation process can enhance the reactor design and improve the elimination of persistent organic pollutant (POP) formation. POPs mainly include substances such as polycyclic aromatic hydrocarbons (PAHs), polychlorinated dibenzo-p-dioxins (PCDDs), and polychlorinated dibenzofurans (PCDFs) [20]. Primary pyrolysis and subsequent reaction of dominant volatile compounds are essential stages for producing POPs during the thermal degradation [17]. According to Luda et al., the degradation products obtained from PP pyrolysis can be explained by a mechanism associated with random scission followed by intramolecular H transfer [21]. On the other hand, researchers under the leadership of Ma suggested that the intramolecular transfer of secondary radicals play an essential role in the thermal degradation of PP [18].

Even before the COVID-19 pandemic outbreak, plastic waste management was considered a major environmental issue due to growing concerns about global pollution. Nevertheless, to deal with the increased production of disposable face masks, we need to determine their degradation and flammability characteristics for efficient waste management. Moreover, it has been recognized that the proper management of used PPE waste plays a vital role in preventing the further spreading of COVID-19 [22]. Methods based on oxygen depletion measurements such as pyrolysis combustion flow calorimetry have been proven to provide reliable results [23]. Pyrolysis is considered one of the best waste management methods compared to other thermal treatments, as it is effective in diminishing the carbon footprint of plastic wastes [24]. Hence, in our report, we focus on the characterization of individual parts of the masks, made of different materials, and assessment of their thermo-oxidative degradation as well as the pyrolysis of single-use face masks via FTIR, TG, and MCC techniques.

## 2. Materials and Methods

### 2.1. Materials

In this work, commercially available disposable face masks were purchased from different manufacturers. Prior to analysis, they were cut into small samples, which are shown in Figure 1. Figure 1a shows a multi-layer mask with an FFP3 breathing valve produced by OXYLINE sp. z o.o., Pabianice, Poland. For this mask, samples were taken from the center of the fabric (M-1A), face strap (M-1B), and breathing valve (M-1C). Figure 1b shows a simple, white, three-layer mask made by the melt-blown method and produced by 4Mass S.A., Warszawa, Poland. For this mask, samples were taken from the center of the fabric (M-2A) and face strap (M-2B). The last and most popular type of mask is presented in Figure 1c. It is a surgical mask made in Guangzhou, China by Guangzhou Xinzhou Health company. For this mask, samples were also taken from the center of the fabric (M-3A) and face strap (M-3B). 

### 2.2. Methods

#### 2.2.1. Fourier Transform Infrared Spectra (FTIR)

Fourier transform infrared spectra (FTIR) were recorded using the Thermo Scientific spectrophotometer model Nicolet iS5 (Thermo Fisher Scientific, Carlsbad, CA, USA), operating in an attenuated total reflectance mode (ATR) with a C/ZnSe crystal. Each measurement range was 4000–450 cm^−1^, with a scan number of 16 and resolution of 4 cm^−1^.

#### 2.2.2. Thermal Analysis

The thermogravimetric analysis was performed under air atmosphere using a Netzsch TG 209 F1 Libra thermogravimetric analyzer (Netzsch, Selb, Germany). The measurements were conducted in the temperature range from 30 to 600 °C at a heating rate of 10 °C/min in the synthetic air atmosphere with an airflow rate of 25 cm^3^/min. Sample mass was kept in the range of 4.50–4.60 mg, measured in open α-Al_2_O_3_ crucibles.

In addition, measurements were carried out in an inert atmosphere (nitrogen) in the temperature range from 30 to 600 °C at a heating rate of 30 °C/min in order to compare the results of thermal analysis with the measurements made by Microscale Combustion Calorimetry (MCC).

#### 2.2.3. Pyrolysis Combustion Flow Calorimetry

Pyrolysis properties were also tested through Microscale Combustion Calorimetry (MCC) using a PCFC Fire Testing Technology Ltd. (Fire Testing Technology, East Grinstead, UK) analyzer according to ASTM D7309 method A at a synthetic air mixture volume ratio of 80/20 (nitrogen/oxygen). The mass of the samples was ca. 5 mg and the heating rate was 30 °C/min. The studies were conducted within the temperature range of 100–750 °C.

Based on the procedure proposed in [25], for TG and MCC data, the reaction rates were calculated using Formulas (1)–(3):

(1) $$\dot{r_{m}}=-\left(dm/dt\right)/\left(m_{0}-m_{\infty }\right)$$

(2) $$\dot{r_{q}}=\dot{q}/\bar{∆q^{\prime }}$$

(3) $$∆q^{\prime }=\dot{q}/\dot{r_{m}}$$

where

$\dot{r_{m}}-$ the reaction rate of weight loss, s^−1^;

dm/dt− weight derivative over time;

$m_{0}-$ the initial mass of the sample, kg;

$m_{\infty }-$ the final mass of the sample, kg;

$\dot{r_{q}}-$ the reaction rate of heat release, s^−1^;

$\dot{q}-$ specific heat release rate, W/g;

$∆q^{\prime }-$ the heat of combustion per unit mass of the sample, J/g;

$\bar{∆q^{\prime }}-$ total heat of combustion per unit mass of the sample, J/g.

## 3. Results and Discussion

### 3.1. FTIR Analysis

Disposable face masks are manufactured using various polymers and inorganic additives, and generally, there is no available detailed information on their composition [1]. For this reason, it is necessary to characterize the types of used materials by, e.g., the FTIR technique, before further analysis of the thermal and flammability behavior. The resulting FTIR spectra of face mask parts are shown in Figure 2.

The comparison of the absorbance band distribution on the FTIR spectra of the M-1A, M-1C, M-2A, and M-3A samples showed identical bands in the two broad ranges from 2835 to 2952 and from 1165 to 1452 cm^−1^, which is characteristic for the FTIR spectrum of polypropylene (PP) [26]. The FTIR spectrum showed four large bands in the wavenumber range 3000–2800 cm^−1^; the bands at 2950 and 2865 cm^−1^ were attributed to CH_3_ asymmetric and symmetric stretching vibrations, respectively, while the bands at 2915 and 2865 cm^−1^ were due to CH_2_ asymmetric and symmetric stretching vibrations, respectively [27]. The FTIR spectrum also showed two intense bands at 1452 and 1375 cm^−1^, caused by CH_3_ asymmetric and symmetric deformation vibrations, respectively [28]. The band at 1165 cm^−1^ could be attributed to C–C asymmetric stretching, CH_3_ asymmetric rocking, and C–H wagging vibrations [28]. Results of IR analysis indicate that all three masks were made of polypropylene sheets.

The mask strap M-1B was composed mainly of poly(ethylene terephthalate) fiber and a thin inner rubber band; the FTIR spectrum is shown in Figure 2a. The analysis of the FTIR database showed the similarity of the tested material with the spectrum of ethylene propylene diene rubber (EPDM) filled with talc—often used as a filler for various types of rubbers and mineral oil. The latter component is added during the mixing of rubber with fillers to improve the flow characteristics [29]. In the spectrum of EPDM, the broad band at 3385 cm^-1^ was assigned to O-H stretching vibration [30]. This band also appears in the talc spectrum, attributed to the surface hydroxyl groups [31]. The band at 2917 cm^−1^, present in both EPDM and talc spectra, was assigned to the asymmetric stretching vibration of the methylene asymmetrical stretching band. The band at 2850 cm^−1^ originated from the symmetric stretching vibration of the methylene group in EPDM [30]. The characteristic peak at 1595 cm^−1^ was assigned to unsaturated carbon-carbon bond stretching vibration. The bands at 1447 cm^−1^ and 1375 cm^−1^ were assigned to -CH_2_- scissoring vibration and symmetric C-H stretching vibration, respectively. The band at 1030 cm^−1^ could be ascribed to the symmetric vibration of carbon-oxygen-carbon or the stretching vibrational bands of siloxane group from talc [31], whereas the band at 3676 cm^−1^ could be assigned to the vibrations of OH groups linked with Mg; the band at 671 cm^−1^ corresponded to the Si-O-Mg bond in talc filler [31].

Ear strap samples M-2B and M-3B exhibited identical FTIR spectra to polyamide 6 [32]. The molecular structure of polyamide 6 consists of amide groups (CO-NH) separated by linear chains of methylene units [-(CH_2_)_5_-], and all amide groups are oriented approximately perpendicular to the polymer chain axis and form intermolecular hydrogen bonds [32]. The N-H stretching region of polyamides occurs in the range of about 3100–3500 cm^−1^ [33]. Around 3300 cm^−1^, a distinct absorption band appeared related to hydrogen-bonded NH stretching; band 3062 cm^−1^ was associated with NH Fermi resonance and band 2926 cm^−1^ correlated with asymmetric and 2856 cm^−1^ with symmetric CH_2_ stretching vibrations [32]. Primarily due to the carbonyl stretching vibration, the amide I band occurred at 1631 cm^−1^ and the amide II band at 1533 cm^−1^. The characteristic absorption bands were also 1460 cm^−1^ and 1414 cm^−1^ (CH_2_ scissors vibration), 1364 cm^−1^ (amide III and CH_2_ wag vibration), 1198 cm^−1^, and 1257 cm^−1^ (CH_2_ twist-wag vibration) [33,34].

### 3.2. Thermogravimetric Analysis

A thermogravimetric experiment under the oxidative atmosphere was performed before the pyrolysis study to analyze the thermo-oxidative degradation profiles of the disposable face mask. The samples’ mass losses and decomposition temperatures are given in Table 1, while the thermo-oxidative degradation curves are shown in Figure 3.

The data presented in the table and the graph confirm that M-1A, M-1C, M-2A, and M-3A samples are made of the same material, as they show thermal degradation characteristic of polypropylene. A two-stage thermo-oxidation profile characterizes PP. The TG curve of the M-3A sample has a slightly different course. The curve slope is less steep, which shows that the degradation rate is lower for this face mask. The final decomposition temperature (T_endset_) is higher by about 30 degrees than other samples, which may indicate that stabilizing additives were used in this face mask [1]. Indeed, the residue at 600 °C is considerably bigger in this sample than in the rest of the PP mask parts. It is noteworthy that pristine polypropylene decomposes into a large number of aliphatic compounds without a residue [35].

Similar but not identical thermograms characterize the ear strap of the first two face masks (samples M-1B and M-2B). The curves show a three-stage thermo-oxidative degradation of samples. Initial decomposition temperature (T5%) varies slightly between 332 °C and 340 °C. Significant differences are revealed after comparing maximum degradation peaks in all of the decomposition stages. The first stage appears in the temperature range of 270–380 °C, with the peaks’ maxima at 370 °C (M-1B) and 315 °C (M-2B). The second step appears between 380 and 460 °C, and the maxima of peaks occur at 426 °C and 411 °C, respectively. The last, third step takes place between 480 and 550 °C, with the peaks’ maxima at 506 °C and 528 °C, respectively.

Three very distinct stages of decomposition characterize the ear strap of the third face mask (M-3B). The pristine PA6 exhibits single-stage degradation, with DTG maximum at 452 °C, which may indicate that we are not dealing with a pure polymer [36]. The first stage appears around 300–365 °C, with the maximum DTG peak at 330 °C. The biggest second step occurs around 280–480 °C, with a maximum of 452 °C. The last step starts at about 540 °C and ends above 600 °C. The mass of the solid residue, which is still 4.1% of the initial mass, indicates lower flammability.

### 3.3. Pyrolysis Combustion Flow Calorimetry

Figure 4 shows the Heat Released Rate (HRR) plots as a function of temperature for samples obtained from the middle (central) part of the mask (Figure 4a) and the mask mount (Figure 4b).

The presented diagrams show that the primary material from which the masks are made, regardless of its origin (Figure 4a), burned quite rapidly in a one-step process in the range from 350 to 520 °C in 166 s. The rapid burning of these samples is evidenced by the steep course of the curves, which can be observed for all of the pieces. Slight differences can be found in peak heat release rate (PHRR) values, which were noted as 1129 W/g (479 °C), 1175 W/g (477 °C), and 1190 W/g (476 °C) for M-1A, M-2A, and M-3A, respectively.

On the other hand, a slightly different trend was observed for the tested masks’ mount burning process. In the case of sample M-1B, the combustion process proceeded in at least three stages, with visible maxima at 344 °C (43 W/g), 387 °C (270 W/g), and 442 °C (288 W/g). This indicates the complexity of the synthetic material of the fastener, which is more fire-resistant than the main mask material. The complexity of the M-1B material also suggests that compounds formed during its decomposition at lower temperatures may accelerate the other compounds’ thermal degradation.

In the M-2B sample, a three-stage combustion process was observed, with the first peak recorded at 317 °C and the next ones at 431 °C and 453 °C. This may mean that a small admixture of a compound with the lowest activation energy is burned first. Then, substances, similar in terms of their flammability, are incinerated in the subsequent steps. The nature of the changes of the peaks within the temperature range of 380–520 °C suggests the occurrence of parallel, sequential degradation reactions. Comparing M-1B and M-2B samples, it should be noted that no differences were observed in the case of the number of characteristic peaks and PHRR values, which were, in fact, very similar to each other. This fact confirms the previous conclusions obtained from the FTIR study that M-1B and M-2B mask straps are made of the same material. The differences were concentrated in the appearance of these peaks at different temperatures and with different total heat release (THR) values. The M-1B sample was 43.6 kJ/g, and the M-2B sample was 16.1 kJ/g.

Sample M-3B burned in an entirely different, multi-step way. The curve was characterized by a gradual increase in the heat release rate, in the range of 280–410 °C, thus suggesting the complexity of the decomposition process in this temperature range. Further heating to 510 °C reveals at least two stages: the first at 446 °C (307 W/g), and the second with a maximum at 468 °C (474 W/g). Thus, we cannot find any similarities with the combustion mechanisms observed for the M-1B and M-2B samples but rather with the M-3A sample. The decomposition of the M-3B sample reaches a temperature of 540 °C, which means that this sample burns for the longest time of all tested samples, i.e., for 517 s.

Based on the calculations of the reaction rates, graphs comparing the TG and MCC analyses were drawn (Figure 5). High compliance of the reaction rate curves calculated based on TG and MCC data was obtained for the samples as shown in Figure 5a–c. A slight shift in the maximum values of the reaction rate as a function of temperature may result from different process conditions for TG and MCC analysis (shapes of chambers, gas flow rate). The comparison of the curves shows that most of the sample mass is lost at the temperature corresponding to the heat release maximum during the main decomposition stage of samples M-1A, M-2A, and M-3A. The analysis presented in Figure 5 shows that the decomposition rate is slow in the temperature range of 200–400 °C, and heat is released close to 5 kJ/g. In addition, the volatile substances released during the main decomposition stage have a low calorific value (approximately 6.1 kJ/g for M-1A, 5.7 kJ/g for M-2A, and 6.6 kJ/g for M-3A), while most flammable, volatile substances (with the heat of combustion above 30 kJ/g) are formed at higher temperatures (above 550 °C). It is worth noting that the total heat of combustion, which is 41.06, 43.61, and 44.24 kJ/g for M-1A, M-2A, and M-3A, respectively, differs from the calculated values by 9.74, 9.72, and 7.03 kJ/g, respectively.

In the results presented in Figure 5d–f, changes in the reaction rate distribution are more complicated. Most of the mass of sample M-1B is lost at a temperature close to that where the second heat release occurs. For this sample, a similar two-stage reaction rate increment is maintained, suggesting either the presence of at least two different materials or the overlapping of at least two major decomposition reaction mechanisms. In samples M-2B and M-3B, the range of heat release rate corresponds to the rate of mass loss. In addition, for these two samples in the range of 200–400 °C, the heat of combustion is released with a value not exceeding 5 kJ/g, and the decomposition reaction rate is prolonged. The volatile substances released during the primary decomposition step have a calorific value of approximately 1.4 kJ/g for M-2B and 1.1 kJ/g for M-3B. In addition, in the case of these samples, a large proportion of the flammable, volatile substances are formed at temperatures above 550 °C.

Nevertheless, the calculated values of the heat of combustion are lower than those presented in Figure 3. The experimental THR value for the M-2B sample was 16.08 kJ/g, and for the M-3B sample, 28.80 kJ/g. This may suggest that both the masks and their mounts were made of similar materials, with a similar decomposition mechanism. The situation observed in the case of the M-1B sample decomposition requires a separate comment. The heat of combustion of this mask mount in the range of 200–400 °C exceeds the value of 5 kJ/g and is characterized by two maxima at a temperature of approximately 246 °C (13.22 kJ/g) and 377 °C (7.06 kJ/g). In terms of the occurrence of maximum losses of mass and heat release (i.e., in the temperature range 280–520 °C), the calorific value of volatile substances is also tiny. On the other hand, a sharp increase in the calorific value occurs in the final stage of afterburning of the char, i.e., temperatures above 520 °C. This is also confirmed by experimental data in the form of THR equal to 81.06 kJ/g.

## 4. Conclusions

The sudden increase in single-use masks during the COVID-19 pandemic underlines the crucial need for a proper disposal method, so they do not end up in landfills, posing a hazard.

The comparison of the absorbance band distribution on the FTIR spectrum of the M-1A, M-1C, M-2A, and M-3A samples shows identical bands in the two broad ranges from 2835 to 2952 cm^−1^ and from 1165 to 1452 cm^−1^, which is an FTIR spectrum characteristic of polypropylene (PP). This indicates that all three masks were made out of polypropylene sheets, which is the major component of waste. Ear straps M-2B and M-3B exhibited various FTIR peaks with polyamide 6, and M-1B was mainly composed of poly(ethylene terephthalate) fiber and thin inner EPDM rubber filled with talc and mineral oil.

The thermogravimetric analysis showed decomposition stages and temperatures for all samples. The thermal degradation mechanism of polypropylene fits perfectly to that presented by the M-1A, M-1C, M-2A, and M-3A samples. All mount strap samples show three stages of degradation, but with a different course of decomposition profile. The maximum degradation of the first stage varies, being 315 °C, 330 °C, and 370 °C for M-2B, M-3B, and M-1B, respectively. The M-1B ear strap left the highest residue and is expected to exhibit the lowest flammability among all samples.

Summarizing the MCC analysis, M-2 and M-3 masks and their attachments burn relatively quickly, all in a very similar way, generating heat at the level of 45 kJ/g. Considering that both parts are made out of polypropylene, a non-charring polymer, they are fully decomposed during calorimetry. On the other hand, the M-1 mask has a mask mount made of a much less bulky material than the central part of the mask, and when burning, this part of the mask generates twice as much heat as the central part itself.

The analysis of flammability and thermogravimetric results show that the most heat is generated above 450 °C, where the main combustion stage practically disappears for some materials, as was the case for M-1B and M-2B. Therefore, to ensure that the thermal utilization of single-use mask waste is effective while maintaining proper energy management, it should be carried out in the temperature range from 450 to 750 °C.

## Figures and Tables

**Figure 1:** Photos of the face masks and sample denotation: (**a**) multi-layer mask with an FFP3 breathing valve; (**b**) three-layer mask made by the melt-blown method; (**c**) surgical mask made in China.

**Figure 2:** FTIR spectra of different parts of disposable face masks: (**a**) multi-layer mask with an FFP3 breathing valve; (**b**) three-layer mask made by the melt-blown method; (**c**) surgical mask made in China.

**Figure 3:** Thermo-oxidative degradation of different parts of disposable face masks: (**a**) TG and (**b**) DTG profiles of center parts of the fabrics and the valve; (**c**) TG and (**d**) DTG profiles of the face straps, respectively.

**Figure 4:** The heat release rate dependence as a function of temperature for samples (**a**) M-1A, M-2A, and M-3A and (**b**) M-1B, M-2B, and M-3B.

**Figure 5:** The dependence of the reaction rate and the heat of combustion as a function of temperature for the samples (**a**) M-1A; (**b**) M-2A; (**c**) M-3A; (**d**) M-1B; (**e**) M-2B; (**f**) M-3B. HRR—Heat Released Rate; TG—thermogravimetric analysis; HoC—Heat of combustion.

**Table 1:** Mass losses and decomposition temperatures of all samples.

Sample Denotation	T_5%_ (°C)	T_onset_ (°C)	T_endset_ (°C)	T_max1_ (°C)	T_max2_ (°C)	T_max3_ (°C)	Residue at 600 °C (%)
M-1A	263	278	332	316	448	-	0.4
M-1B	332	349	529	370	426	506	9.5
M-1C	267	278	328	315	497	-	1.5
M-2A	267	282	330	317	465	-	0.3
M-2B	340	379	552	315	411	528	2.4
M-3A	264	276	360	324	483	-	2.4
M-3B	320	312	471	330	452	557	4.1

## Data Availability

Data is contained within the article.
